This article has been retracted.

# Ranking candidate genes of esophageal squamous cell carcinomas based on differentially expressed genes and the topological properties of the co-expression network

**DOI:** 10.1186/s40001-014-0052-x

**Published:** 2014-10-29

**Authors:** Yuzhou Shen, Jicheng Tantai, Heng Zhao

**Affiliations:** Department of Thoracic Surgery, Shanghai Chest Hospital, Shanghai Jiao Tong University, 241 Huaihai (West) Rd, Shanghai, 200030 People’s Republic of China

**Keywords:** Esophageal squamous cell carcinomas, Differentially expressed genes, Topological properties, Co-expression network, Candidate genes

## Abstract

**Background:**

The aim of this study was to identify the candidate genes of esophageal squamous cell carcinoma (ESCC).

**Methods:**

Gene expression profiling of 17 ESCC samples and 17 adjacent normal samples, GSE20347, was downloaded from Gene Expression Omnibus database. The raw data were preprocessed, and the differentially expressed genes (DEGs) between ESCC and normal samples were identified by using SAM software (false discovery rate <0.001). Then, the co-expression network of DEGs was constructed based on Pearson’s correlation test (r-value ≥0.8). Furthermore, the topological properties of the co-expression network were analyzed through NetworkAnalyzer (default settings) of Cytoscape. The expression fold changes of DEGs and topological properties were utilized to identify the candidate genes of ESCC (Cri_n_ score >4), which were further analyzed based on DAVID functional enrichment analysis (*P*-value <0.05).

**Results:**

A total of 1,063 DEGs were identified, including 490 up-regulated and 573 down-regulated DEGs. Then, the co-expression network of DEGs was constructed, containing 999 nodes and 46,323 edges. Based on the expression fold changes of DEGs and the topological properties of the co-expression network, DEGs were ranked, and the top 24 genes were candidate genes of ESCC, such as *CRISP3*, *EREG*, *CXCR2*, and *CRNN*. Furthermore, the 24 genes were significantly enriched in bio-functions regarding cell differentiation, glucan biosynthetic process and immune response.

**Conclusion:**

The present study suggested that *CRISP3*, *EREG*, *CXCR2*, and *CRNN* might be causative genes of ESCC, and play vital roles in the development of ESCC. However, further experimental studies are needed to confirm our results.

**Electronic supplementary material:**

The online version of this article (doi:10.1186/s40001-014-0052-x) contains supplementary material, which is available to authorized users.

## Background

Esophageal squamous cell carcinoma (ESCC) is the predominant histologic subtype of esophageal cancer, which is characterized by high mortality rate and geographic differences in incidence [1]. ESCC is a common malignant cancer worldwide, especially in China [2]. Recently, clinical therapies have been used to treat ESCC, such as neoadjuvant chemoradiotherapy [3,4], surgery [5], and combination therapy [6]. However, these approaches do not increase survival rate of patients with ESCC. To investigate novel therapies, a clear understanding of the molecular pathogenesis of ESCC is required, to which much effort has been made.

Microarray analysis has been widely used to investigate gene expression in various diseases, such as breast tumors [7], brain cancer [8], endometrial cancer [9], and renal cell carcinoma [10]. In previous studies of ESCC, loss of heterozygosity (LOH) and copy number alteration in ESCC were identified by using microsatellite markers and low- and high-density SNP arrays [11,12]. The differentially expressed genes (DEGs) and microRNAs between ESCC and normal squamous epithelia have been identified based on microarray analysis [13,14]. Moreover, a comprehensive survey of commonly inactivated tumor suppressor genes in ESCC was performed based on microarray analysis and functional reactivation of silenced tumor suppressor genes by 5-aza-2′-deoxycytidine and trichostatin [15]. Thus, microarray analysis is a useful approach to identify key genes involved in ESCC.

In our study, microarrays were utilized to identify the DEGs between human ESCC samples and adjacent normal tissues samples. Then, the co-expression network of DEGs was constructed, and the topological properties of the co-expression network were analyzed. Additionally, we built an integrated index to rank DEGs and identify the candidate genes of ESCC. Furthermore, the relevant functions of candidate genes were investigated. We anticipate that our work can find key genes related with ESCC, and provide new insights for target therapies.

## Methods

### Microarray data and preprocessing

The raw gene expression profile GSE20347 [2] was downloaded from the public functional genomics database Gene Expression Omnibus (GEO, http://www.ncbi.nlm.nih.gov/geo/). In total, 34 specimens were available, including 17 human ESCC samples and 17 matched adjacent normal tissues samples. None of the patients with ESCC had received prior therapy, and informed consent was obtained. Demographic and clinical information were matched. The corresponding platform was GPL571, [HG-U133A_2] Affymetrix Human Genome U133A 2.0 Array. The background correction and normalization of microarray data among chips were conducted based on RMA (Robust Multiarray Averaging) method [16]. When several probes were mapped to one gene, their mean value was taken as the gene expression value of this gene.

### DEG screening

SAM 4.0 software [17] was used to screen out the DEGs between ESCC and normal samples. SAM is a widely used tool for DEG screening. The criterion for this analysis was false discovery rate (FDR) <0.001.

### Hierarchical clustering analysis of DEGs

To determine the specificity of DEGs between ESCC and adjacent normal samples, the pheatmap package in R was utilized to perform bidirectional hierarchical clustering analysis (BHCA) [18,19]. Rationally, after BHCA, ESCC and adjacent normal samples are supposed to be distinguished clearly by DEGs.

### Constructing the co-expression network of DEGs

In organisms, biological functions are often based on the interaction of several genes, and significantly co-expressed genes are usually co-regulated and involved in the same or similar biological processes and pathways [20]. In order to identify the co-expressed DEGs in ESCC tissues, the expression values of DEGs in each sample were abstracted, and Pearson’s correlation test was used to calculate the correlation coefficient (r-value) of DEGs. Higher *P*-value represents stronger correlation between node ‘n’ and its adjacent nodes, and only the co-expressed DEG pairs with r-value ≥0.8 were utilized to construct the co-expression network of DEGs, which was visualized by using Cytoscape [21].

### Analyzing the topological properties of the co-expression network

The topological properties (node degree and clustering coefficient) of DEGs in the co-expression network were analyzed based on NetworkAnalyzer of Cytoscape software [22]. Node degree and clustering coefficient are important topological properties of network. Node degree ‘k_n_’ is the number of nodes connected to node ‘n’, displaying the local centrality of this node in network. Higher node degree represents stronger importance of a node for the stability of network. Clustering coefficient of node ‘n’ is defined as:

$$ {\mathrm{C}}_{\mathrm{n}}=2{\mathrm{e}}_{\mathrm{n}}/\left[{\mathrm{k}}_{\mathrm{n}}\left({\mathrm{k}}_{\mathrm{n}}\hbox{-} 1\right)\right] $$

In this formula, ‘k_n_’ is the number of adjacent nodes, and ‘e_n_’ is the number of interconnections among adjacent nodes. Representing the clustering degree of node ‘n’, C_n_ is between 0 and 1, and higher C_n_ represents that the adjacent nodes of node ‘n’ connected with each other more closely.

### DEG ranking and candidate gene identification

Candidate genes of ESCC could be identified by ranking DEGs based on expression fold changes, node degrees, and clustering coefficients in the co-expression network. In this study, firstly, Z-transformation was performed to transform three sets of data into Z-scores, which are common standardized scores in statistics [23]. Secondly, the ranking index of each DEG was calculated based on the formula as follows:

1 $$ \mathrm{C}\mathrm{r}{\mathrm{i}}_{\mathrm{n}}=\mathrm{F}{\mathrm{C}}_{\mathrm{n}}+\mathrm{degre}{\mathrm{e}}_{\mathrm{n}}+\mathrm{C} $$

Here, Cri_n_ is the ranking index of gene ‘n’, FC_n_ is the expression fold change of gene ‘n’, degree_n_ is the node degree of gene ‘n’ in theco-expression network, and C_n_ is the clustering coefficient of gene ‘n’ in the co-expression network. Thirdly, the DEGs with Cri_n_ score >4 were defined as candidate genes of ESCC.

### Functional enrichment analysis

To reveal the biological process associated with ESCC, gene ontology (GO) functional enrichment analysis was performed for the candidate genes of ESCC based on the Database for Annotation, Visualization and Integrated Discovery (DAVID) [24]. DAVID provides exploratory visualization tools to promote functional classification. In this study, the criterion for this analysis was a *P*-value <0.05.

## Results

### Identification of DEGs and hierarchical clustering analysis

After preprocessing and DEG screening, 1,063 DEGs (FDR <0.001) were identified between ESCC and adjacent normal samples, including 490 up-regulated and 573 down-regulated DEGs. After BHCA, ESCC and adjacent normal samples could be distinguished clearly by DEGs (Figure 1).

**Figure 1:** **Bidirectional hierarchical clustering analysis of differentially expressed genes.** The green to red gradation represented the changes of expression value from down-regulation to up-regulation.

### Construction of the co-expression network

The r-values of DEG pairs were calculated based on Pearson’s correlation test, and the co-expression network of DEGs with r-value ≥0.8 were constructed (Additional file 1). The co-expression network involved 999 nodes (DEGs) and 46,323 edges (co-expression relationships), and it was further divided into two closely connected large sub-networks.

### DEG ranking and candidate gene identification

To identify the candidate genes of ESCC, we established an integrated ranking index by integrating the expression fold changes, node degrees, and clustering coefficients of DEGs in the co-expression network. Consequently, a total of 24 genes were candidate genes (Cri_n_ score >4) of ESCC (Table 1), such as cysteine-rich secretory protein 3 (*CRISP3*), epiregulin (*EREG*), chemokine receptor 2 (*CXCR2*), and cornulin (*CRNN*).

**Table 1:** **The 24 candidate genes of esophageal squamous cell carcinomas**

**Rank**	**Symbol**	**Rank**	**Symbol**
1	*CRISP3*	13	*CYP4B1*
2	*EREG*	14	*SLURP1*
3	*ENDOU*	15	*MAL*
4	*CXCR2*	16	*TGM3*
5	*CRCT1*	17	*CWH43*
6	*FLG*	18	*TMPRSS11E*
7	*CLIC3*	19	*CLCA4*
8	*CRNN*	20	*PPP1R3C*
9	*MMP1*	21	*BBOX1*
10	*GYS2*	22	*HPGD*
11	*EPB41L3*	23	*SPINK5*
12	*SCEL*	24	*FCER1A*

### Functional enrichment analysis

To understand the biological processes involving candidate genes, GO functional enrichment analysis (*P*-value <0.05) was performed. It was found that the 24 candidate genes were significantly enriched in bio-functions regarding cell differentiation, glucan biosynthetic process and immune response, including epidermal cell differentiation, epithelial cell differentiation, epidermis development, keratinocyte differentiation, glucan biosynthetic process, and regulation of immune response (Table 2).

**Table 2:** **Functional enrichment analysis of the 24 candidate genes**

**GO ID**	**GO term**	***P*** **-value**
GO:0009913	Epidermal cell differentiation	2.43E-06
GO:0030855	Epithelial cell differentiation	3.14E-05
GO:0008544	Epidermis development	9.93E-05
GO:0030216	Keratinocyte differentiation	1.10E-04
GO:0008544	Epidermis development	1.21E-04
GO:0007398	Ectoderm development	1.34E-04
GO:0060429	Epithelium development	2.23E-04
GO:0009888	Tissue development	1.15E-02
GO:0009250	Glucan biosynthetic process	1.70E-02
GO:0005978	Glycogen biosynthetic process	1.70E-02
GO:0033692	Cellular polysaccharide biosynthetic process	3.54E-02
GO:0050776	Regulation of immune response	4.14E-02
GO:0044042	Glucan metabolic process	4.87E-02
GO:0006073	Cellular glucan metabolic process	4.87E-02
GO:0009913	Epidermal cell differentiation	2.43E-06
GO:0030855	Epithelial cell differentiation	3.14E-05

GO: gene ontology; ID: identifier.

## Discussion

In the present study, we identified 1,063 DEGs between ESCC and adjacent normal samples, including 490 up-regulated and 573 down-regulated genes. Furthermore, the co-expression network of DEGs was constructed, consisting of 2 large sub-networks, 999 nodes, and 46,323 edges. Then, the expression fold changes, node degrees, and clustering coefficients of DEGs in the co-expression network were comprehensively analyzed to rank DEGs, and 24 candidate genes of ESCC were identified.

Among the 24 candidate genes, the highest ranking was *CRISP3*. It was originally discovered in human neutrophilic granulocytes, and is a glycoprotein that belongs to a family of cysteine-rich secretory proteins (CRISPs) [25]. In previous studies, *CRISP3* is found to be overexpressed in prostate adenocarcinoma by using quantitative real-time reverse-transcription-PCR [26]. Additionally, Su *et al*. reveal that *CRISP3* is significantly down-regulated in ESCC, and may be the biomarker of ESCC [27]. Furthermore, *CRISP3* was reported to be down-regulated in oral squamous cell carcinoma (OSCC), and the loss of its DNA copy number was observed in two of the five OSCC-derived cell lines [28].

*EREG* was the second highest ranking of 24 candidate genes whose protein product, EREG, induces cell growth by binding to the epidermal growth factor receptor (EGFR) [29]. It is reported that *EREG* is epigenetically silenced in gastric cancer cells by aberrant DNA methylation and histone modification [29]. Moreover, EREG is involved in the invasion and metastasis of esophageal carcinoma by combining with sphingosine kinase-1 (SPHK1) [30].

*CXCR2*I codes a receptor of ELR + CXC chemokines, which are potent promoters of angiogenesis [31]. It is reported that GROA-C XCR2 and GROB-C XCR2 signaling contribute significantly to esophageal cancer cell proliferation, and this autocrine signaling pathway may be involved in esophageal tumorigenesis [32,33].

*CRNN* codes cornulin, a Ca^2+^ − binding protein that presents in the upper layer of squamous epithelia [34]. It has been shown that the large majority of ESCC cases have little or no expression of cornulin in carcinoma or stromal cells [35]. These evidences suggested that *CRISP3*, *EREG*, *CXCR2*, and *CRNN* may play crucial roles in ESCC, as well as other candidate genes.

In addition, GO functional enrichment analysis was performed, and some biological processes were enriched significantly, such as epidermal cell differentiation, epithelial cell differentiation, epidermis development, keratinocyte differentiation, and regulation of the immune response. It has been shown that proliferation and development of esophageal epithelial cells are associated with the development of ESCC [36]. Moreover, ESCC-related gene modules are significantly enriched in epidermal cell differentiation, epithelial cell differentiation, epidermis development, and keratinocyte differentiation [37]. Additionally, keratinocytes migrate from the basal to the superficial layers of the epidermis, and undergo morphological and biochemical changes during terminal differentiation, which are involved in the development of ESCC [38,39]. Our results were consistent with these evidences.

## Conclusions

In conclusion, the DEGs between ESCC and adjacent normal tissues were screened out, and the co-expression network was constructed, consisting of 2 large sub-networks, 999 nodes, and 46,323 edges. After analyzing the gene expression and topological properties of DEGs in the co-expression network, DEGs were ranked, and 24 candidate genes of ESCC were identified. Candidate genes, such as *CRISP3*, *EREG*, *CXCR2*, and *CRNN*, were identified as potentially playing key roles in the development of ESCC. Furthermore, functional enrichment analysis revealed that the 24 genes were mainly enriched in epithelial cell differentiation, epidermis development, and keratinocyte differentiation. These results provided us with candidate genes and demonstrated their potential functions in the development of ESCC. However, more experimental studies are needed to confirm these results.

## Additional file

Additional file 1:
**The co-expression network of differentially expressed genes.**
